RETRACTED

# The Value of CBL-Based Teaching Mode in Training Medical Students' Achievement Rate, Practical Ability, and Psychological Quality

**DOI:** 10.1155/2022/2121463

**Published:** 2022-08-26

**Authors:** Yaying Zhao, Wenfang Liu, Zhemin Wang, Xinglin Chen, Jinying Zhao, Xianbo Zhou

**Affiliations:** ^1^18 Ward, Hangzhou Lin'an District First People's Hospital, Hangzhou 311300, China; ^2^20 Ward, Hangzhou Lin'an District First People's Hospital, Hangzhou 311300, China

## Abstract

In order to improve the quality of medical student training, the clinical case-based learning (CBL) teaching mode is analyzed in the aspect of the rate of achievement, practical ability, and psychological effect. A total of 86 medical students who came to our hospital from March 2020 to December 2021 are selected and divided into the CBL group and the control group according to the random number table method. The psychological quality of medical students is evaluated by observing their movements and expressions during their internship. In addition, the questionnaire is used to evaluate the scores of a medical student in future planning, occupational health, and teamwork spirit. The compliance evaluation results show that CBL teaching mode can significantly improve the compliance rate of medical students in training and promote the confidence of future role change to a certain extent.

## 1. Introduction

As a discipline focusing on clinical practice and rigor, clinical medicine is closely related to the whole process of patient diagnosis and treatment [1]. An excellent clinician often needs to accumulate a lot of theoretical basis and practical experience in order to make a more accurate diagnosis and treatment of patients [2]. The growth of excellent clinicians is inseparable from the training of high-efficiency medical students. Therefore, applying clinical knowledge to medical practice through scientific and efficient teaching mode plays an important role in the transformation of the role of medical students [3]. At present, the commonly used teaching concepts in clinical practice include problem-based learning (PBL) and research-based learning (RBL). The two teaching modes mentioned above have stimulated the subjective initiative of medical students from different angles and improved their ability to find and deal with problems. However, there are still some defects in the cultivation of practical ability [4, 5]. With the continuous development of medical education, the traditional teaching mode has been unable to meet the diverse learning needs. Case teaching is a new teaching mode developed on the basis of PBL. By guiding teachers to strengthen theoretical knowledge learning in clinical practice, students' practical ability is improved and their comprehensive quality can be further improved [6]. However, there are relatively few studies on the application of CBL in the cultivation of medical students. Therefore, this study selected 86 medical students who practiced in our hospital from March 2020 to December 2021 and adopted different teaching and training methods to observe the impact of CBL on the success rate, practical ability, psychological quality, and other comprehensive qualities of medical students. This study will lay a theoretical foundation for the training of professional clinicians.

RETRACTED

This paper is organized as follows: Section 2 discusses the related work, followed by the teaching mode and assessment methods in Section 3. In Section 4, the results and analysis are presented. Finally, in Section 5, some concluding remarks are made.

## 2. Related Work

With the gradual development of medical education, clinical practice needs to adopt a variety of payment methods to meet different educational needs [7]. Among them, PBL and RBL are the most common teaching modes. Some scholars have suggested that although PBL can enable students to collect information and conduct case analysis by themselves, it can cultivate students' independent ability to solve problems to a certain extent [8]. It can improve students' learning interest in dealing with clinical diseases and give full play to their subjective initiative, so that students play a leading role in teaching [9]. However, we still need to adhere to the evaluation of teaching progress and teaching effect in the teaching process. Unreasonable teaching design or failure to raise questions to the teaching guidance team in time will have a certain impact on the teaching quality [10]. Therefore, CBL is gradually promoted on the basis of PBL. Abstract theoretical knowledge needs to be transformed into practical cases that are easy to understand based on clinical practice. This can not only help medical students consolidate basic knowledge but also combine it with clinical practice [11]. Thus, learning can be transformed into a positive process and relevant knowledge can be effectively mastered.

Relevant research shows that medical students who adopt CBL teaching mode have better psychological quality after practice [12]. CBL mode adopts a practice oriented teaching method to combine actual cases with teaching materials in clinical application [13]. We make medical students have a more vivid and vivid understanding of theoretical knowledge in the learning process, so as to mobilize their subjective initiative in learning. At the same time, different departments explain to students by combining actual cases and guide learning problems by combining theoretical knowledge. It can not only promote the teaching quality in the process of practice but also conduct case analysis through guiding problems. In addition, we summarize and review the key cases to effectively form a pre-memory process for the diagnosis and treatment of the disease [14]. Selective teaching of special and rare cases through CBL teaching mode can improve the ability of medical students to deal with urgent problems. Internship teachers conduct targeted explanations through course demonstrations to achieve various teaching purposes of combining practice with theoretical knowledge [15, 16]. Therefore, the application of CBL mode can enhance practical ability, promote professional development, and enhance team spirit. Further, we promote CBL to give full play to the subjective initiative of medical students, so as to integrate into professional roles faster and to promote the transformation of roles and careers [17, 18]. CBL teaching mode is also conducive to cultivating medical students' exploration spirit and innovation ability. By analyzing the relevant contents of clinical cases and participating in group discussions, medical students can understand and master relevant theoretical knowledge and operational skills [19].

RETRACTED

## 3. Teaching Mode and Assessment Methods

### 3.1. Teaching Mode

The control group uses conventional teaching mode. It mainly includes the following contents: during the admission internship, according to the teaching process of the conventional departments of our hospital, medical students should learn and investigate theoretical knowledge, train and learn in their respective departments, and conduct supplementary teaching of skill chain and theoretical knowledge during the internship.

CBL group adopts clinical case-based learning for teaching, specifically includes: (1) set up a special teaching group with professional doctors as teaching teachers and the teachers of each group completed teaching guidance and operation training for medical students [20]; (2) typical cases with common clinical manifestations are selected for medical students to learn based on their major and teaching content, and the selected cases should have detailed diagnosis and treatment process and complete clinical data [21]; (3) the teacher should combine the questions with the materials and clinical practice, design representative teaching questions, and ask the medical students to look up relevant information within a specified time [22]. If necessary, the teacher should give some guidance and help the medical students to get familiar with the basic situation of the case; (4) during clinical ward rounds and diagnosis and treatment, medical students should be asked to watch and learn, and then the clinical data, general information, imaging data, laboratory examination results, and other indicators of patients are introduced in detail, and relevant questions are put forward for students to think and solve by themselves [23, 24]; (5) carry out group discussion, summarize problems encountered in clinical events into PPT for report, and discuss with other medical students to solve [25, 26]; and (6) during the group discussion of medical students' practice, the teacher shall be responsible for the analysis of important points, give reasonable guidance to the direction, depth and breadth of the discussion of medical students, and check and fill up the gaps. Finally, the medical students' individual summary is made to cultivate the ability of medical students to deal with problems alone, study independently and work in a team [27].

RETRACTED

### 3.2. Assessment Methods

#### 3.2.1. General Information

A total of 86 medical students who came to our hospital for internship from March 2020 to December 2021 are selected and divided into a CBL group and a control group according to the random number table method, with 43 cases in each group. The comparison of baseline data between the two groups is shown in Table 1, indicating comparability (*P* > 0.05).

The inclusion criteria are as follows: (1) good communication and understanding skills; (2) no truancy or truancy occurs; (3) good compliance with teaching; and (4) all students can conscientiously complete the learning tasks assigned by the teacher.

The exclusion criteria are as follows: (1) accompanied by mental diseases; (2) serious absenteeism records during school; (3) disobey the guidance of the teacher; and (4) cheating during the examination.

#### 3.2.2. Assessment of the Compliance Rate

At the end of the internship, students will be comprehensively evaluated in terms of a written test, practical operation, emergency problem solving, and teamwork ability. Teachers in each group will score jointly <60 points will be regarded as unqualified and ≥60 points will be regarded as qualified.

#### 3.2.3. Practical Ability Assessment

The teachers assessed the practical operation ability of medical students in different periods of internship. The observation mainly included proficiency, error rate, emergency handling ability, and completion time. The score is ranged from 0 to 100 and the higher the score, the stronger the practical ability of medical students.

#### 3.2.4. Psychological Quality Assessment

In practice, the teachers in each group observed the psychological quality of medical students in the process of practice by observing their adaptability, cognitive characteristics, personality quality, and other aspects. The score range is 0 to 100 points, and the higher the score is, the stronger the psychological quality of medical students in the process of practice.

RETRACTED

#### 3.2.5. Questionnaire Preparation

At the end of the teaching, the future career planning, team spirit, practical operation ability, and mastery of theoretical knowledge of the two groups of medical students are evaluated through a questionnaire designed by our hospital. The number of medical students is investigated according to the classification of very helpful, uncertain, and unhelpful.

### 3.3. Technical Roadmap

The technical roadmap is shown in Figure 1.

### 3.4. Statistical Processing

SPSS 25.0 statistical software is used for data analysis, and the main factors include the following: (1) Measurement data: If the data followed normal distribution and homogeneity of variance after normality test, they are represented by mean ± standard deviation. Paired sample *T* is used for an intragroup test, variance comparison is used between groups, and repeated measure variance analysis is used for intergroup comparison at various time periods, and spherical test is performed. (2) Count data: descriptive statistical analysis is conducted by percentage, and *χ*^*2*^ test is performed. All the above data showed significant differences with *P* < 0.05.

## 4. Results and Analysis

### 4.1. Comparison of Compliance Rates

At the end of the internship, the assessment of the compliance rate of the two groups of medical students showed that the compliance rate of the CBL group is 39 (90.70%) and that of the control group is 31 (72.09%) (*x*^*2*^ = 4.914, = 0.027). The results suggest that the CBL teaching mode can significantly improve the compliance rate of the training of medical students.

### 4.2. Changes in Practical Ability

The results showed that the practical ability of the two groups of medical students is poor before the practice, and the practical ability is improved after different modes of teaching (*P* < 0.05). Compared with the control group, the time ability level of the CBL group is significantly higher in the middle and late stage (*P* < 0.05), as shown in Table 2 and Figure 2. The symbol “*∗*” means that compared with T1, ^*∗*^*P* < 0.05; “&” means ^&^*P* < 0.05 compared to *T*2. Moreover, the “*a*, *b*, *c*” in Figure 2, respectively, means that if the same letter is shared between groups, *P* > 0.05 at different time points.

### 4.3. Psychological Quality Assessment

The psychological quality of the students in each group is evaluated by the teachers during the practical operation, and the results showed that the psychological quality of CBL patients is significantly better than that of the control group (*P* < 0.05) as shown in Table 3 and Figure 3.

RETRACTED

### 4.4. Future Planning Survey Results

The results showed that there are significant differences between the CBL group and the control group in vocational help, role change promotion, clinical practice ability, and team spirit (*P* < 0.05) as shown in Table 4.

## 5. Conclusions

In this study, the clinical case-based learning (CBL) teaching mode is analyzed in the aspect of the rate of achievement, practical ability, and psychological effect. A total of 86 medical students are selected and divided into the CBL group and the control group according to the random number table method. The control group adopts the conventional teaching mode and the CBL group is applied the CBL teaching mode. The changes of practical ability in early (T1), middle (T2), and late (T3) learning are compared between the two groups. In the process of practice, teachers can evaluate the psychological quality by observing the movements and expressions of medical students. After teaching, a questionnaire is conducted to investigate the scores of medical students on future planning, career fitness, and teamwork spirit. After the internship, the compliance rate of the two groups of medical students is evaluated. The compliance rate of the CBL group is 39 (90.70%) and that of the control group is 31 (72.09%) (*χ*^*2*^ = 4.914, *P*=0.027). The two groups of medical students have poor practice ability before practice, but their practice ability improves after different modes of teaching (*P* < 0.05). Compared with the control group, CBL group can obtain significantly higher level of time ability in the middle and late stage (*P* < 0.05). The psychological quality of CBL patients is significantly better than that of the control group (*P* < 0.05). The results show that there are significant differences between the CBL group and control group in vocational help, role change promotion, clinical practice ability and team spirit (*P* < 0.05). The results indicate that the CBL teaching model can effectively improve the success rate of medical students and improve the clinical practice ability and psychological quality effectively. CBL also can promote the medical students in the professional role of resilience and improve the team cooperation spirit.

## Figures and Tables

**Figure 1:** Technology roadmap.

**Figure 2:** The changing trend of each group's practical ability.

**Figure 3:** Contrast of psychological quality.

**Table 1:** The baseline data.

	CBL group (*n* = 43)	Control group (*n* = 43)	*t/χ* ^*2*^	*P*
Age (years)	23.11 ± 1.52	23.18 ± 1.31	−0.229	0.820
*Gender*			0.048	0.826
Man	26 (60.47%)	25 (58.14%)		
Woman	17 (39.53%)	18 (41.86%)		
BMI (kg/m^2^)	22.31 ± 2.36	22.29 ± 2.4)	0.039	0.969
*Major*			0.084	0.728
Orthopedics department	18 (41.86%)	16 (37.21%)		
Gynecology department	14 (32.56%)	17 (39.53%)		
Stomatology department	11 (25.58%)	10 (23.26%)		

RETRACTED

**Table 2:** Change of practical ability.

Group	*n*	T1	T2	T3	*F*	*P*
CBL group	43	61.23 ± 5.62	73.13 ± 6.42^*∗*^	81.24 ± 6.72^*∗*&^	4.571	<0.001
Control group	43	60.39 ± 5.94	68.73 ± 6.03^*∗*^	75.67 ± 7.41^*∗*&^	3.581	<0.001
*t*		0.674	3.276	3.651		
*P*		0.502	0.002	<0.001		

**Table 3:** Contrast of psychological quality.

Group	*n*	Psychological quality
CBL group	43	76.45 ± 6.52
Control group	43	64.45 ± 8.93
*t*		7.117
*P*		<0.001

**Table 4:** Future planning survey results.

Item	CBL group (*n* = 43)			Control group (*n* = 43)			*χ* ^*2*^	*P*
	Helpful	Normal	Did not help	Helpful	Normal	Did not help		
Help your future career	34	9	0	24	11	8	0.083	<0.001
Team work spirit	37	6	0	22	15	6	0.031	<0.001
Clinical practice ability	35	7	1	21	18	4	0.052	<0.001
Role change resilience	39	4	0	27	10	6	0.074	<0.001
Communicate ability	34	5	4	32	7	4	0.172	0.535
The emergency ability	31	6	6	30	8	5	0.119	0.617

## Data Availability

The simulation experiment data used to support the findings of this study are available from the corresponding author upon request.
